# Assessment of Load Manual Lifting among Shelf-Stoking Workers in Chain Stores: A Cross-Sectional Study

**DOI:** 10.1155/2024/2324416

**Published:** 2024-01-17

**Authors:** Alireza Choobineh, Elahe Dortaj, Mohsen Razeghi, Haleh Ghaem, Hadi Daneshmandi

**Affiliations:** ^1^Research Center for Health Sciences, Institute of Health, Shiraz University of Medical Sciences, Shiraz, Iran; ^2^Department of Ergonomics, School of Health, Shiraz University of Medical Sciences, Shiraz, Iran; ^3^Department of Physiotherapy, School of Rehabilitation Sciences, Shiraz University of Medical Sciences, Shiraz, Iran; ^4^Department of Epidemiology, School of Health, Shiraz University of Medical Sciences, Shiraz, Iran

## Abstract

In Iranian stores, shelf workers, in addition to shelf-stocking, perform diverse tasks, such as working as a cashier, cleaning, barcode reading, labeling goods, and entering the price with the portable data terminal (PDT). Therefore, this study aimed to investigate the prevalence of work-related musculoskeletal symptoms (WMSs) and assess load manual lifting among shelf-stoking workers. This cross-sectional study was conducted among 101 shelf-stoking workers (60 males and 41 females) in chain stores at Shiraz city, Iran. The subjects were selected by cluster sampling from chain stores in Shiraz city, namely Refah, Canbo, Soroush, and Tirazis. Then, the required number of samples was selected and entered into the study from each cluster in proportion. The Persian version of the Nordic Musculoskeletal Questionnaire and the National Institute of Occupational Safety and Health–variable lifting index method were used to collect the required data. Data were analyzed by SPSS software version 22 using the Mann–Whitney *U* test, Spearman's correlation coefficient, and linear regression. Ankles/feet, lower back, and knees had the highest prevalence of WMSs among the participants. About 70.3% of workers had a VLI higher than 1. There was an association between gender and VLI. The VLI was higher in males than females. The study's findings revealed that the medians of the VLI were significantly different among participants with/without upper back symptoms during 12 months prior to the study and among participants with/without lower back symptoms during 7 days prior to the study. According to the linear regression analysis, gender and lower back symptoms during 7 days prior to the study remained in the model and were associated with the VLI. The findings revealed that the back region of the shelf-stoking workers is prone to work-related musculoskeletal disorders. In addition, based on the results, gender and lower back symptoms during the 7 days prior to the study were predicting variables for VLI. This study provides an overview of pain/discomfort and postural load in shelf-stoking workers. Since the principles of ergonomics for the placement and layout of shelves are the same in all stores, the findings of the present study can be used in other stores.

## 1. Introduction

A chain store consists of two or more retail stores with the same management selling the same lines of goods. In chain stores, workers do different jobs, one of which is shelf-stocking. Individuals who work on shelf-stocking tasks are called shelf or shelf layout workers [1, 2].

Manual lifting task is an important part of daily duties for shelf-stock workers. After unloading trucks, workers carry loads, place them inside the shelves, and transfer the remaining to the warehouse. All of these operations are done manually and often without assistive devices. Usually, shelf workers deal with different weights of loads and put them at different heights [2].

Studies have shown that lifting loads from different heights affects the body biomechanically [3, 4]. One research in Italy showed that biomechanical stress was high for retailers with lifting tasks [5]. Silvetti et al.'s [4] study conducted on shelf workers of grocery stores by electromyography, and the National Institute for Occupational Safety and Health (NIOSH) equation showed that shelf height had a significant effect on biomechanical parameters and stress on the musculoskeletal system.

In shelf-stocking, manual handling is inevitable that exerts a high force on the back [6]. In this case, the cost of related injuries such as low back pain (LBP) is considerable [7, 8]. Violante et al. [2] reported the prevalence of 12-month LBP in the fruit and vegetable section of the supermarket as 34.5%. In addition, previous studies have shown that there is an association between LBP and high physically demanding jobs such as load lifting [9, 10], individual characteristics such as age, body mass, and gender [11], as well as psychological demands [12].

There is little epidemiological data on work-related musculoskeletal disorders (WMSDs) among shelf workers [4]. In 2001, of 180,000 work-related injuries and illnesses in the U.S. industry, 42,600 were related to individuals working in the grocery stores [13]. Based on the literature, about 50%, 10%, and 6% of LBP are related to lifting, pushing and pulling, and carrying loads, respectively [14].

In ergonomics, there are many methods, such as the NIOSH equation, the Washington Industrial Safety and Health Act (WISHA) checklist, the 3D Static Strength Prediction Program (3DSSPP), etc., for assessing the load manual lifting [15]. Studies carried out by Dempsey et al. in 2005 [16] and 2019 [17] showed that the NIOSH equation was the most common observational method used by ergonomists to evaluate manual lifting. Besides, Waters et al. [18] described four classifications of lifting: (a) single-task manual lifting, (b) multiple-task manual lifting, (c) sequential manual lifting, and (d) variable-task manual lifting. The shelf-stoking task is of the fourth type.

It should be noted that the results of the Bosch et al. [19] study indicated that although there were other methods for manual lifting than NIOSH, such as Composite Lift Index (CLI), Sequential Lifting Index (SLI), and Variable lifting index (VLI), 83%, 86%, and 89% of evaluators were not aware of these methods, respectively.

The idea for the method of VLI evaluation is similar to the technique of CLI for the composite task. The contrast is that instead of utilizing a single task component, all lifts will first be aggregated into a maximum of 30 subtasks and the corresponding Frequency-Independent Lifting Index (FILI), which will then be divided into a fixed number of FILI categories (e.g., six), each with a variable frequency. Then, these six FILI groups will be weighted (3) using the CLI equation.

Most ergonomic research in large-scale stores has been carried out on cash registers [20, 21].

In Iran, shelf workers, in addition to shelf-stocking, perform diverse tasks, such as working as a cashier, cleaning, barcode reading, labeling goods, and entering the price with the portable data terminal (PDT).

Given the above, we carried out the present study to determine the prevalence of work-related musculoskeletal symptoms (WMSs) and evaluate load manual lifting in shelf workers.

## 2. Materials and Methods

### 2.1. Study Population and Sample Selection

In this cross-sectional study, after a general review of chain stores in Shiraz city, Iran, four chain stores were selected for the following reasons: (a) they were part of the large chain stores in Shiraz, (b) the staff of these stores had shelf-stocking duties, (c) the shelf-stocking tasks in these stores were relatively similar, (d) the workers did shelf-stocking tasks for at least 2 hr a day, and (e) the stores had more than four branches in Shiraz city.

According to statistics, the total number of shelf-stocking workers in the chain stores in Shiraz city was 485. The number of samples was calculated using the below formula. Considering a 20% loss, 101 shelf-stoking workers (60 males and 41 females) were investigated in the study. The mean ± standard deviation of height, weight, age, work experience, and body mass index (BMI) were 170.5 ± 8.6 cm, 69.3 ± 13.3 kg, 27.3 ± 4.6 years, 3.4 ± 2.9 years, and 23.7 ± 3.7 kg/m^2^, respectively.

(1) $$\begin{array}{c} n=\frac{Z_{1-\frac{\alpha }{2}}^{2}pq}{d^{2}}=\frac{1.96^{2}\times 0.3\times 0.7}{0.1^{2}}=81, \end{array}$$

where *Z*^2^ = 1.96 for a significant level of 5%, *d* = 0.1, *p* (prevalence of WMSs) = 0.3, *q* (1 − *p*) = 0.7.

The data were extracted from the study of Violante et al. [2].

Male and female workers were included in the study as per their percentages in the target population. Furthermore, these individuals were selected by cluster sampling from these stores so that the selected individuals had a balanced distribution with no bias. In this study, clusters four were public chain stores in Shiraz city, namely Refah, Canbo, Soroush, and Tirazis. Then, the required number of samples was selected and entered into the study from each cluster in proportion.

Inclusion criteria were employees working in chain stores with a shelf-stocking job and having at least 1 year of work experience in age ranging from 18 to 45 years, while exclusion criteria included the presence of musculoskeletal disorders (MSDs) that had led to an interruption of work for more than a day.

### 2.2. Ethical Considerations

Participants were informed about the study protocol and objectives before the commencement of the study. The participants had a right to withdraw from the study at any time. The study was approved by the ethics committee of Shiraz University of Medical Sciences (Approval ID: IR.SUMS.REC.1398.1129). Additionally, the study was performed in accordance with the Helsinki Declaration of 2013 [22].

### 2.3. Data Collection Tools

The data collection tool in this study consisted of four parts as follows:

#### 2.3.1. Demographic/Occupational Characteristics Questionnaire:

This questionnaire included questions about age, gender, work experience, height, weight, working posture, and the presence of MSDs that led to an interruption of work for more than 1 day.

#### 2.3.2. Persian Version of the Nordic Musculoskeletal Questionnaire (P-NMQ):

The Nordic General Questionnaire was designed and developed in 1987 by Kuorinka et al. [23] by the Scandinavian Institute of Professional Health. The NMQ consists of 18 questions with a dichotomous response (Yes/No) about musculoskeletal symptoms during the last 12 months or the last 7 days. All these questions refer to 9 areas: neck, shoulders, elbows, wrists/hands, upper back, lower back, hips/thighs, knees, and ankles/feet. To facilitate the identification of the anatomical areas, it also includes a body map. This questionnaire has high validity and reliability. Validity tests against clinical history (one study on 19 medical secretaries and one study on 20 railway maintenance workers) showed that the number of nonidentical answers varied between 0% and 20%. Reliability tests with the test–retest method of preliminary versions of the general questionnaire (one study on 29 safety engineers, one study on 17 medical secretaries, and one study on 22 railway maintenance workers) showed that the number of nonidentical answers varied from 0% to 23% [23]. In this study, the P-NMQ was used to examine the reported cases of MSDs among the study population. Cronbach's alpha of this questionnaire in the present study was 0.691.

#### 2.3.3. NIOSH-VLI Equation

In this study, the VLI method developed by Waters et al. [3] was used for evaluation. This method has been validated by Battevi et al. [24]. As the level of VLI increases, the risk of low back injury increases. This risk relationship exists when the VLI is greater than 1 [24].

Also, 1< VLI ≤ 2 is classified as medium risk, 2 < VLI ≤ 3 as high risk, and VLI > 3 as very high risk. The reason for using the VLI method is that the NIOSH lifting equation is more valid than other load-lifting evaluation methods [25]. This method provides a tool to match human abilities with the specific needs of the task [26] and is based on multiple psychophysical, biomechanical, and physiological criteria [27, 28]. To evaluate the fourth type of lifting, the VLI method was used, which was developed by Waters et al. [3] to evaluate jobs with variable load lifting.

The VLI method needs systematic organizational analysis and is focused on a detailed review of the parameters of the lifting task to be determined analytically: (a) The total work time of the variable lifting. (b) The number of lifted items of various weights during this period. (c) The number of employees involved, thus deciding (for one representative employee) the total frequency of lifts (and the corresponding duration scenario). (d) The partial lift frequency for each weight (or group of similar weights). (e) Estimated frequencies of individual lifts according to different lift geometries for identical weights in each group [3].

The parameters mentioned above were obtained by directly observing the workplace, sales data, product sales sites, fixed dimensions such as shelf height and width, and the use of photo and video measurement software such as Digimizer version 6.3.0 [29] and Kinovea version 0.8.15 [30].

In this study, the VLI method of systematic organizational analysis and Colombini simplification methods [25, 31] were used to evaluate shelf tasks.

To obtain more accurate values for the required dimensions in the VLI method, photos and videos were taken from the working environment based on the NIOSH [32] video recording protocol and entered into Digimizer and Kinovea softwares. Then the desired values (dimensions such as H and V) were obtained.

According to the NIOSH imaging protocol [32], a single camera was used for all recordings and was used for at least 10 min for accurate shooting. When filming, we tried to keep a distance of at least 1 m to the subject. Also, it was attempted to film the worker from different directions (front, back, and side) while performing the task for at least 10 min. Besides, if needed, the task was filmed more than once. Photos were also extracted from the recorded videos.

Fixed dimensions such as shelf height and width were measured using a measurement tape.

Figure 1 shows shelf-stoking workers while the load manual lifting.

### 2.4. Statistical Methods

Data analysis was performed by descriptive statistics (frequency and frequency percentage and mean and standard deviation) and analytical statistics (Mann–Whitney *U* test, Spearman's correlation coefficient, and linear regression) using SPSS software version 22. The Mann–Whitney *U* test was used to examine the relationship between VLI with gender and symptoms in different body regions. Spearman's correlation test was applied to study the correlation between VLI with work experience, age, and BMI. Finally, stepwise linear regression was used to examine the simultaneous effects of variables on VLI. Kolmogorov–Smirnov test, histogram, and box plot were used to determine the normality of the collected data. In all tests, *p* ≤ 0.05 was considered as a significant level.

## 3. Results

### 3.1. Demographic/Occupational Details and Nordic Questionnaire

The demographic/occupational characteristics of the participants are presented in Table 1.

In 84% of the stores, there was no place for workers to sit and rest in the workplace, workers were not allowed to sit during working hours, and there was only a place away from work for having lunch or changing clothes. None of the workers used mechanical lifting equipment. In this study, 20% of the chain stores used company sales representatives. These individuals were introduced by a specific brand factory to the store or hired by the store to perform the duties. They were responsible for arranging, transporting, and moving goods of the same particular brand. In 30% of the chain stores, they did not work in just one particular branch but often went to other branches if there were high workloads because of, for example, special sales. Besides, in special situations such as high sales, 5% of the chain stores used rotating shift patterns (morning, evening, and night).

There were instructions for putting goods on the shelf in only one of the chain stores. In 60% of the stores, workers placed products on the shelves according to the weight and quantity of the sales. Shelf picking or shelf-stocking in this study was different, such that 30% of the workers lifted the goods packed in one package, whereas 70% of the workers lifted the goods weighing less than 100 g or more separately.

In 20% of stores, the workers in charge of the branch controlled the number of goods entering the branch daily and continuously according to the amount of sales. They tried to keep the number of goods entering the branch according to the number of sales, but this was sometimes prevented based on some of the chief manager's policies.

Moreover, in these stores, some goods were put on top of the shelves when the warehouse was full or there was not enough space at the time.

Figure 2 shows the distribution of musculoskeletal symptoms in different body regions of the participants. As shown, most musculoskeletal symptoms during the 12 months and 7 days prior to the study were related to the ankles/feet, lower back, and knees.

### 3.2. VLI Analysis

The VLI analysis results are presented in Figure 3. As shown, based on the VLI analysis, most of the workers were put in the “1 < VLI ≤ 2” category, followed by the “0 < VLI ≤ 1” category.

The direct workplace observation data for the VLI calculation showed that the shelves used in the workplace were 130–250 cm high with a depth of 20–100 cm. In these stores, the lowest shelves were 15–50 cm high.

The workers spent the rest of their working hours on warehousing and transportation, cash registering, cleaning, barcode reading, labeling, and pricing with the PDT.

For about 120–160 min per shift, the workers placed products (weighing 30 g–10 kg) on 4–7 shelves. Vertical and horizontal distances were 18–100 cm and 20–100 cm, respectively. In addition, poor grip was observed (CM = 0.90). The mean number of lifted objects per worker per shift was 773.21 ± 456.97.

The mean and standard deviation of the VLI was 1.5 ± 0.9. Also, the lowest and highest VLI values were 0.2 and 3.4, respectively.

The results of the Spearman correlation analysis indicated no significant correlation between VLI and work experience, age, and BMI (*p* ≥ 0.05).

The results of the Mann–Whitney *U* test examine the difference between mean values of VLI in gender groups are depicted in Table 2. As shown, the VLI mean is significantly higher in male workers than the female workers (*p*=0.035).

### 3.3. Association between VLI and Musculoskeletal Symptoms

Table 3 shows that VLI means are significantly different only for groups with/without upper back region symptoms during 12 months prior to the study (*p*=0.045). On the other hand, Table 4 demonstrates that VLI means are significantly different only for groups with/without lower back region symptoms during the 7 days prior to the study (*p*=0.005).

The variables that had *p* < 0.2 in the univariate test were entered into the stepwise linear regression model [33] to investigate the simultaneous effects of variables on the VLI. The variables included in the model were gender, age, height, BMI, working posture, upper back discomfort during the 12 months, and lower back discomfort during the 7 days.

Finally, two variables remained in the model, gender and lower back discomfort during 7 days. The results are presented in Table 5.

According to the linear regression analysis on VLI (Table 5), gender and lower back discomfort during the last 7 days prior to the study remained in the model (*p*=0.012). The model formula is as follows:

(2) $$\begin{array}{c} {\text{VLI}}_{\text{mean}}=1.435+\left(-\text{Lower back }7\text{d}\times 0.480\right)+\left(\text{Gender}\times 0.375\right). \end{array}$$

In this equation, lower back.7d is a back discomfort during 7 days.

According to this equation, the VLI in workers with lower back discomfort in the last 7 days was 0.48 units, which was less than for workers without this discomfort. The regression model also showed that VLI was 0.375 units, higher in females as compared to male workers.

VLI was inversely related to lower back discomfort in the last 7 days but was directly related to gender. As shown in Table 5, the value of adjusted *R* square in this model was 0.069, so about 7% of the changes in VLI could be predicted by gender and lower back discomfort in the last 7 days.

## 4. Discussion

### 4.1. Demographic/Occupational Characteristics and Nordic Questionnaire

The results of the present study indicated that 86.1% of the study workers were young, with an average age of 27.03 ± 4.6 years, and 77.2% had a job experience of fewer than 4 years.

In the present study, workers' posture mainly was standing or kneeling (70%), and in most stores, there was no place for workers to sit and rest.

In Violante et al.'s [2] study, the posture of stocking-shelf workers was 70% standing, 20% kneeling, and 10% walking. Previous studies have shown that prolonged standing causes pressure on the lower back and lower limbs [26, 34]. In addition, Andersen et al. [35] found that standing for more than 30 min at work was a strong predictor of LBP development.

About 71% of the participants had pain and discomfort in at least one body region. MSDs accounted for more than 62% of all occupational health problems in the European transport and storage sector in 2007 [36]. In 2014, about 40% of the reported occupational diseases were in the U.S. warehouses [37]. According to a review study conducted by Asante et al. [38], the 12-month prevalence of LBP is between 16% and 74% in waste collection workers. A survey among freight workers in the central market of India by Gangopadhyay and Das [39] showed that they felt pain and discomfort in all parts of the body.

Furthermore, Forcier et al. [20] indicated that 83% of supermarket workers (excluding cashiers) reported a musculoskeletal disorder for at least the last 12 months. In the study by Violante et al., [2] the 12-month prevalence of LBP was 34.5%, and there was little difference between supermarkets and department stores. In addition, according to a study by Anton and Weeks [40], approximately 78% of grocery store workers reported work-related musculoskeletal disorder symptoms in at least one area of their body, and most workers complained of lower back and leg disorders. And the study by Forcier et al. [20] also reported a high prevalence of WMSDs in supermarket workers, with 83% of the approximately 4,000 workers surveyed (excluding cashiers) reporting a musculoskeletal disorder over 12 months. Furthermore, according to a review study by Azizpour et al. [41] on the prevalence of LBP in 1 year in Iran, the prevalence of LBP in the age group over 24 years with an average of 55.2% (95% CI: 33.7–76.8) was the highest. In this study, the prevalence of LBP in the last 12 months was 23.8%, which could be because 86.1% of the workers were young, with an average age of 27.03 ± 4.6 years. In the Hong et al. [42] study, the prevalence of musculoskeletal discomfort in at least one body region within the past 12 months was 69.1% among manual porcelain workers: the neck (49.3%), lower back (43.8%), and shoulders (27.5%). Hanumegowda et al. [43] reported that about 76.83% of the traditional lacquerware toy makers (77.4% males and 74.28% females) have self-reported WMSDs. In addition, in a systematic review of work-related musculoskeletal disorders among handicraft workers, the findings suggested that the prevalence of musculoskeletal symptoms among handicraft workers is 38.5%–100%, and the most affected body areas were the neck, back, knees, and upper limbs [44].

The reason for the difference in prevalence of musculoskeletal symptoms in our study in comparison to previous studies can be attributed to (1) the difference in the age range of the subjects; (2) the difference in the assessment tools; and (3) the relative difference in the nature of the participants' jobs.

As mentioned before, in the present study, knee and leg discomfort prevalence was high. In the studied stores, the large number of activities performed below knee height was very high due to the low height of shelves. In this situation, workers had to kneel while arranging these shelves with poor posture. In this study, 23% of the workers had a kneeling posture. This may be the reason for the higher prevalence of pain and discomfort in the lower limbs, especially the foot and ankle, in the target workers compared to other parts of the body. Research conducted by Silvetti et al. [4] on greengrocery workers showed that shelf height significantly impacted several parameters, such as knee range of motion (ROM).

The causes of shoulders and hands discomfort in this study might be due to (1) placing objects on shelves higher than the worker's shoulder height, (2) storing some goods on top of the shelves with insufficient space, (3) workers' poor postures due to the depth of the shelf and the placement of objects at the bottom of the horizontal surface of the shelves, and (4) awkward postures of the shoulders and hands due to the use of inappropriate tools and objects as the starting surface to place objects on it and then remove the object and place on the shelf. The finding of the study by Cordeiro et al. [45] indicated that placing loads at a low level compared to the elbow height was a risk factor for MSDs. Likewise, according to a study by Jorgensen et al. [46], placing load-carrying pallets in areas with lower elevations causes bending and twisting of the trunk and shoulders to one side.

### 4.2. VLI

In the present study, 53.5% of the workers had a VLI of 1–2, and 70.3% had a VLI of more than 1. The average value of VLI was 1.5. This indicated that physical stress exerted on the body when lifting the load was high in these workers, which might have caused the back injury, so corrective actions had to be taken as soon as possible. These findings were consistent with a study in Italy by Maso et al. [5] in which the VLI of retailers with lifting tasks was higher than 1. The VLI value of retail workers with manual material handling ranged from 2.12 to 2.811 in the study conducted by Maso [5]. Nicoletti et al. [47] reported that in construction workers, the mean VLI was 2.1; Tirloni et al. [48] also estimated the VLI in slaughterhouse workers with manual material handling to be 4.99. The present study's findings were consistent with the results of these three studies.

Furthermore, according to Battevi et al. [24], the risk of LBP increases as the VLI level increases, which occurs when the VLI is greater than 1. In the present study, the prevalence of LBP in the last 12 months and the last 7 days was 23.8% and 17.8%, respectively. The regression analysis results also showed that the amount of VLI could be predicted with LBP in the last 7 days. As a result, it could be concluded that a reason for the back injury in the subjects was lifting over the limit.

Moreover, as mentioned, the minimum and maximum VLI values in this study were 0.27 and 3.4, respectively. In the Nicoletti et al. [47] study, a research project to assess the risk of manual lifting and carrying in construction companies in the Basilicata area, the minimum and the maximum values of VLI in workers with lifting tasks were also in this range.

In this study, the factors that had the most significant impact on the final VLI were as follows:

- Height coefficient: The height coefficient in the VLI calculation for V bad, which included a height of less than 51 cm and a height of more than 125 cm, was 0.78.
- Horizontal coefficient: The horizontal coefficient in the VLI calculation was 0.71 for H near, 0.56 for H medium and 0.40 for H far.
- Lifting frequency: Lifting frequency significantly affected the VLI [5].
- Weight of lifted objects: The weight of the lifted objects affected the average weight group and eventually the frequency of lifting.

Maso et al. [5] reported that the most important coefficients for reducing VLI were lifting frequency and load weight. In the study performed by Tirloni et al. [48], the amount of VLI in slaughterhouse workers with MMH task was estimated to be 4.99 (very high), but the VLI value was 0.80 and decreased with strategies such as job rotation with eight workers, ideal vertical area, and weight reduction of boxes to 7–8 kg.

As previously mentioned, workers picked up goods weighing less than 100 g separately, which increased the lifting frequency and thus increased the VLI. To reduce the load lifting frequency and consequently to reduce the VLI, these goods can be grouped and packaged with a safe weight. For example, in this study, if workers, who had a VLI of 1.006 and picked goods weighing less than 100 g separately, picked these items in batches, the total frequency value would decrease from 7.743 to 6.66, and consequently, the VLI decreased to 0.895.

### 4.3. The Effect of Variables on Each Other

In the present study, there was a significant relationship between gender and VLI, and according to the regression model, the mean VLI in females was 0.367 units lower than the males. In studies with the VLI method, few comparisons have been made between men and women. Whereas, in studies with the NIOSH equation, the present study results are consistent with the study results by Maina et al. [49]. However, Busto Serrano's findings showed that males are more vulnerable to physical risk factors. In contrast, females seem more affected by psychological risk factors and activities performed outside their working hours. Gender should be considered to ensure the success and effectiveness of ergonomic interventions for the entire working population [50].

Additionally, according to Busto Serrano's study, the variables affecting MSDs are not the same for men and women. In fact, some of the factors associated with physical work limitations explain WMSDs more to men (for example, boring/painful postures, repetitive arm, and hand movements, and heavy handling), while other limitations of physical and mental work explain the symptoms of WMSDs more often in women (for example, lifting or carrying objects, not being able to rest when needed, monotonous work, and work at high speed) [50]. However, in the present study, there were differences between men's and women's load handling tasks, such that men lifted heavier and more loads.

The regression analysis results showed the effect of low back discomfort in the last 7 days on VLI. These results may indicate that since 87.1% of the workers studied were young, with an average age of 27.33 ± 4.968 years old, and 48.5% had less than 2 years of work experience, the cumulative load effects on these workers were not yet evident. Another study by Brauer et al. [51] on airport baggage handlers showed that workers with 20 years of work experience had LBP with a 1.94 incidence rate ratio (IRR) compared to workers with less than 3 years of work experience. The linear correlation of cumulative years of luggage handling with LBP with adjusted IRR 1.16 increased for more than 5 years of work experience [51].

In this study, the amount of VLI was not significantly related to work experience, which could indicate that heavier tasks are usually allocated to workers with less work experience in the workplace, which can cause more VLI in this group [52].

Strengths of the study include (a) considering women in this study, (b) considering shelf-stocking tasks in the chain stores with a highly variable range of lifting dimensions, and (c) performing the highest number of VLI evaluations compared to the previous studies.

However, since this cross-sectional study was conducted in Shiraz and the shelf-stocking job, the results cannot be generalized to other cities or stations.

## 5. Conclusion

The findings of the study revealed that the studied workers' postures were mainly standing or kneeling, and in most stores, there was no place for workers to sit and rest. This may be the one reason for the higher prevalence of pain/discomfort in the lower back, knees, and ankles/feet in the target workers compared to other parts of the body.

VLI analysis indicated that physical stress exerted on the body when lifting the load was high in shelf-stoking workers, which might have caused the back injury. The most important factors for decreasing VLI were found to be lifting frequency, load weight, and height coefficient.

The findings of this study showed the difference between VLI values in women and men, but the regression results indicated that VLI might be predicted by lower back discomfort in the last 7 days and gender in shelf-stocking workers.

This study provides an overview of pain/discomfort and postural load in shelf-stoking workers. Since the principles of ergonomics for the placement and layout of shelves are the same in all stores, the following ergonomic corrective measures and interventions can be recommended for the studied stores and other stores: (a) transferring workers to branches with a higher workload in special circumstances, (b) job rotation, (c) lifting lower weight items together, (d) placing a restraining sheet on the back of the shelf, (e) not placing the items with the lowest sales on the shelves at very low or very high heights, (f) using suitable mechanical devices to move and lift the load, and (g) using lightweight plastic pallets instead of wooden or metal. It is believed that these actions can reduce VLI value and consequently minimize workers' exposure to manual material handling risk factors.

### 5.1. Suggestions for the Future

1. Using other biomechanical assessment methods, such as AnyBody, to evaluate shelf-stoking workers.
2. Conducting more studies on a large scale in this working group.
3. Conducting studies about the impact of organizational issues on this job.

## Figures and Tables

**Figure 1:** Shelf-stoking workers while the load manual lifting.

**Figure 2:** Percentage of musculoskeletal symptoms in different body regions during the 12 months and 7 days prior to the study (*n* = 101).

**Figure 3:** The result of the variable lifting index (VLI) analysis among the studied workers (*n* = 101).

**Table 1:** Some personal details of the workers studied (*n* = 101).

Variable	Number	Percent
Gender		
Male	60	59.4
Female	41	40.6
Height (cm)		
<160	12	11.9
160–170	42	41.6
>170	47	46.5
Weight (kg)		
<50	3	3.0
50–70	60	59.4
>70	38	37.6
Age (years)		
<20	7	6.9
20–30	80	79.2
>30	14	13.9
Body mass index (kg/m^2^)		
<18	3	3.0
18–25	68	67.3
>25	30	29.7
Work experience (years)		
<2	39	38.6
2–4	39	38.6
>4	23	22.8
Working posture		
Walking	30	29.7
Standing	48	47.5
Kneeling	23	22.8

Mean ± standard deviation of height, weight, age, work experience, and BMI were 170.5 ± 8.6 cm, 69.3 ± 13.3 kg, 27.3 ± 4.6 years, 3.4 ± 2.9 years, and 23.7 ± 3.7 (kg/m^2^), respectively.

**Table 2:** Comparison of the median of the variable lifting index (VLI) among gender groups of the workers studied (*n* = 101).

Gender	VLI ^*∗*^	*P* value^†^
	Median (IQR ^*∗∗*^)	
Male (*n* = 42)	1.67 (1.01, 1.73)	0.035
Female (*n* = 59)	1.27 (0.50, 1.41)	
Total (*n* = 101)	1.5 ± 0.9	—

^*∗*^Variable lifting index.  ^*∗∗*^Interquartile range. ^†^Mann–Whitney *U* test.

**Table 3:** Comparison of the median of the variable lifting index (VLI) in workers with/without symptoms in different body regions during 12 months prior to the study (*n* = 101).

Body region	VLI ^*∗*^		*P* value^†^
	With symptom	Without symptom	
	Median (IQR ^*∗∗*^)	Median (IQR ^*∗∗*^)	
Neck	1.398 (1.237, 1.974)	1.378 (0.508, 1.724)	0.295
Shoulders	1.418 (0.923, 1.725)	1.378 (0.508, 1.724)	0.523
Elbows	1.725 (1.004, 2.379)	1.378 (0.816, 1.724)	0.243
Wrists/hands	1.398 (0.985, 1.725)	1.378 (0.508, 1.724)	0.763
Upper back	1.725 (1.172, 3.033)	1.378 (0.508, 1.721)	0.045
Lower back	0.715 (0.410, 1.725)	1.398 (1.006, 1.724)	0.161
Hips/thighs	1.571 (0.628, 1.725)	1.378 (0.852, 1.724)	0.693
Knees	1.418 (1.122, 1.725)	1.378 (0.498, 1.724)	0.228
Ankles/feet	1.375 (0.504, 1.724)	1.398 (0.923, 1.724)	0.686

^*∗*^Variable lifting index,  ^*∗∗*^Interquartile range, ^†^Mann–Whitney *U* test.

**Table 4:** Comparison of the median of the variable lifting index (VLI) in workers with/without symptoms in different body regions during 7 days prior to the study (*n* = 101).

Body region	VLI ^*∗*^		*P* value^†^
	With symptom	Without symptom	
	Median (IQR ^*∗∗*^)	Median (IQR ^*∗∗*^)	
Neck	1.544 (1.378, 3.270)	1.378 (0.644, 1.724)	0.164
Shoulders	2.110 (0.565, 3.280)	1.378 (0.852, 1.724)	0.632
Elbows	1.451 (1.013, 2.101)	1.378 (0.781, 1.724)	0.15
Wrists/hands	1.146 (0.688, 2.383)	1.388 (0.816, 1.724)	0.73
Upper back	1.671 (0, 1.006)	1.378 (0.712, 1.724)	0.485
Lower back	0.501 (0.370, 1.454)	1.398 (1.146, 1.724)	0.005
Hips/thighs^††^	—	—	—
Knees	1.705 (0.725, 2.472)	1.378 (0.852, 1.721)	0.097
Ankles/feet	1.006 (0.453, 1.685)	1.398 (0.937, 1.724)	0.137

^*∗*^Variable lifting index,  ^*∗∗*^Interquartile range, ^†^Mann–Whitney *U* test, ^††^Missing data.

**Table 5:** Linear regression model indicating factors with an influence on variable lifting index (VLI) (*n* = 101).

Model	*R* ^*∗*^	*B* ^*∗∗*^	SE^†^	Beta	*T* ^††^	Sig.	Adjusted *R* square
Gender	0.214	0.375	0.176	0.206	2.136	0.035	0.069
Lower back symptoms during 7 days prior the study	0.297	−0.480	0.225	−0.206	−2.133	0.035	

^*∗*^Coefficient of determination.  ^*∗∗*^Unstandardized beta coefficient. ^†^Standard error. ^††^*T*-distribution.

## Data Availability

The data used to support the findings of this study are available from the corresponding author upon request.
